The article "Region Dual Attention-Based Video Emotion Recognition" was published in 2022. Journal: Comput Intell Neurosci.

# Region Dual Attention-Based Video Emotion Recognition

**DOI:** 10.1155/2022/6096325

**Published:** 2022-06-15

**Authors:** Xiaodong Liu, Huating Xu, Miao wang

**Affiliations:** School of Computing, Henan University of Engineering, Zhengzhou, China

## Abstract

To solve the emotional differences between different regions of the video frame and make use of the interrelationship between different regions, a region dual attention-based video emotion recognition method (RDAM) is proposed. RDAM takes as input video frame sequences and learns a discriminatory video emotion representation that can make full use of the emotional differences of different regions and the interrelationship between regions. Specifically, we construct two parallel attention modules: one is the regional location attention module, which generates a weight value for each feature region to identify the relative importance of different regions. Based on the weight, the emotion feature that can perceive the emotional sensitive region is generated. The other is the regional relationship attention module, which generates a region relation matrix that represents the interrelationship of different regions of a video frame. Based on the region relation matrix, the emotion feature that can perceive interrelationship between different regions is generated. The outputs of these two attention modules are fused to produce the emotional features of video frames. Then, the features of video frame sequences are fused by attention-based fusion network, and the final emotion feature of the video is produced. The experimental results on the video emotion recognition data sets show that the proposed method outperforms the other related works.

## 1. Introduction

Emotion plays a very important role in people's daily life. Emotional intelligence is to be considered an important part of human intelligence. With the continuous improvement of people's demand for intelligence, emotional intelligence, which is an important part of human intelligence has attracted extensive attention in the field of artificial intelligence [1]. Although the intelligent computer has become a part of human life, the relationship between human and machine is stiff and lacks emotional communication. If the machine can understand the human emotional state, it will provide more comfortable service. Emotion recognition is an important part of comprehensive understanding of video scenes. It is the key technology of intelligent security, human-computer interaction, and video recommendation. Video emotion recognition technology has become one of the hot issues in the field of computer vision.

The traditional video emotion recognition method is based on manual features. It learns the mapping relationship between emotion features and emotion types through pattern classifier and rule reasoning. De Silva and Ng [2] construct a facial expression recognition system based on video temporal features and a hidden Markov model based on audio features. However, the accuracy of video emotion recognition based on low-level manual features is relatively low. In recent years, with the success of the convolutional neural network (CNN) in the field of image classification and object detection, researchers try to use CNN to improve the accuracy of emotion recognition. In paper [3], CNN is used to analyze image emotion. The results show that the accuracy of the CNN feature is better than manual low-level features. Human emotion is expressed through multiple modes, some researchers extract the features of multiple modes by CNN, and then these features are fused to establish multimodal video emotion features. Chen et al. [4] extract multimodal features from audio and visual modes, further improving the performance of video emotion recognition, which means the complementarity between different modes. Kim and Provost [5] use the average features of the upper face, lower face, and speech signals to obtain the final emotion label. This average aggregation strategy cannot reflect the differences in video emotion expression. Due to the differences in face size, posture, perspective, and the emotional differences contained in context, the amount of emotional information contained in different video frames is also different.

The article "Region Dual Attention-Based Video Emotion Recognition" was published in 2022. Journal: Comput Intell Neurosci.

The attention mechanism allows people to focus on useful information while ignoring irrelevant signals and noise. In recent years, it has been widely used in the field of computer vision. Some researchers [6, 7] use the attention network to generate a weight for each video frame. The video frames are fused according to their weight to make full use of the information differences between different video frames. In recent studies, attention-based video emotion recognition has attracted more and more attention. Emotional expression may only appear in some scenes. Barros et al. [8] use convolutional neural networks to learn the location of emotional expression in video frames. Lee et al. [9] propose a spatiotemporal attention network, which can selectively locate the targeted emotional regions from a long speech spectrogram. In these researches, the attention mechanism is mainly used to solve the emotional differences between different video frames.

However, due to the diversity of human emotional expression, the emotional expression is also different in different regions of the same video frame. Human emotional expression is not limited to the face. Poses and gestures may also contain rich emotional clues and the emotional information contained in different parts are also different. In addition, the video frame may also contain contextual information such as scenes and objects, which also contain different emotional clues. When we judge the emotion of a video frame, we often focus on the areas that contain rich emotional clues. As an example, take a look at the images in Figure 1. Let us try to estimate what they feel. In Figure 1(a), the human face and posture contain more emotional clues. It is easier to identify the human emotions in the video frame by focusing on the areas of these two parts. Similarly, detailed estimations method can be made in other figures of Figure 1. Therefore, how to make full use of the emotional clues of different regions of the video is a significant challenge for video emotion recognition.

The article "Region Dual Attention-Based Video Emotion Recognition" was published in 2022. Journal: Comput Intell Neurosci.

There are not only emotional differences but also mutual relations between different regions of the video. The relation of some regions is close, which will make it easier to recognize human emotions in video frames. For example, in Figure 1(c), the combination of the human face, human arm, and dog can more easily recognize human emotion. However, the relationship between some regions is relatively loose, and the combination of these regions is not helpful for emotion recognition.

The existing emotion recognition methods extract the emotional features of the whole video frame, which may contain faces, different parts of the human, scenes, and objects. These features are finally transformed into a unified emotional representation through full connection operation, which cannot effectively express the relationship between different regions. Therefore, how to establish the relationship between different regions is another challenge for video emotion recognition.

To overcome the above two challenges, this paper proposes a region dual attention-based video emotion recognition method (RDAM). It takes as input the video frames to learn a discriminative video emotion representation that can solve the emotional differences of different regions and make full use of the relationship between different regions. The main contributions of this paper are as follows:

1. This paper proposes a video emotion feature extraction method based on the regional dual attention mechanism. It consists of two parallel attention modules: one is the regional location attention module, which generates a weight for each region to identify the relative importance of different regions. The emotion features are recalculated based on the generated weight to generate the features of perceptible emotion sensitive regions. The other is the regional relationship attention module, which generates a regional relationship matrix representing the relationship between any two regions. The emotional features are recalculated according to the regional relationship matrix, and the emotional features which can perceive the interrelationship between regions are obtained. Finally, the outputs of the two attention modules are fused to further improve the representation of emotional features.
2. A video frames feature fusion method is proposed, which fuses features of the video frames when the emotional features of each video frame are generated by the region dual attention module. It also uses the attention mechanism to obtain the emotional weight of video frames and fuses the features of video frames according to their emotional weight to generate the emotional features of the video.

The article "Region Dual Attention-Based Video Emotion Recognition" was published in 2022. Journal: Comput Intell Neurosci.

We have carried out experimental verification on video emotion recognition data sets. The experimental results show that the region dual attention mechanism can focus on emotion sensitive regions and make full use of the relationship between regions, to improve the accuracy of video emotion recognition.

## 2. Related Works

### 2.1. Feature-Fusion-Based Emotion Recognition

Human emotion is often expressed through multiple modes. The human face, audio, human body, action, and environment are all contain emotional clues. Integrating emotional clues of multiple modes can further improve the performance of emotion recognition. The experiments of the paper [10] show that when fusing context and body information, the performance is better than that using only body or context information. MCEF [11] models human emotion from three complementary aspects: facial appearance, facial movement, and audio. Chen et al. [12] first compute the semantic features of events, objects, and scenes based on CNN. The extracted high-level features are used as emotion context information and are further integrated with a context fusion network to generate a unified representation for video emotion recognition. Vielzeuf et al. [13] propose a hierarchical method that allows the fusion of scores and features in different layers. It can retain different module information when using different module features. These methods improve the performance of video emotion recognition by fusing features of multiple modes, but the time evolution of emotion expression is not considered.

Some researchers model the temporal evolution features of emotion by converse 3d (C3d), long short-term memory (LSTM), or recurrent neural network (RNN). Ye et al. [14] extract audio features with CNN and capture the temporal evolution of intonation by RNN to recognize emotion. Pini et al. [15] fuse static facial features, dynamic evolution of human expression, and audio features. The static facial features and dynamic evolution features of human expression are, respectively, extracted by CNN and C3d, and the time evolution of audio features is extracted by LSTM. These features are fused through a fusion network to form a unified representation. Fan et al. [16] combine CNN-recurrent neural network (RNN) and C3d in a late-fusion fashion. RNN takes as input appearance features extracted by CNN and encodes motion features. C3d model appearance and motion of video simultaneously. These features are combined to generate the representation of the video. Ebrahimi Kahou et al. [17] combine CNN and RNN to recognize emotion. The features of images are first extracted by CNN, and these features are used as RNN input to generate the whole video emotion feature. Fonnegra and Diaz [18] use CNN and RNN to model the temporal and spatial features of facial regions. The convolution layer is used to analyze the spatial information changes of short-time periodic, and the RNN layer is used to model the changes of frames as time-varying time series. Then these layers are connected to multilayer perceptrons to perform classification tasks. However, these features are independent of each other and are emotional cues of different modes. The relationship between different modes has not been considered.

The article "Region Dual Attention-Based Video Emotion Recognition" was published in 2022. Journal: Comput Intell Neurosci.

To establish the relationship between different modes, Mo et al. [19] propose a novel feature set called HHTC features based on the combination of Hilbert–Huang transform (HHT). It is based on the visual features, HHT-based audio features, and cross-correlation features. In addition to the dependencies between the visual and the audio signals, HHTC features also can indicate the time-varying features of these signals. Xue et al. [20] propose a Bayesian nonparametric multimodal data architecture to learn emotions in the video. CNN is used to extract the appearance features of key frames, and Mel Frequency Cepstrum Coefficient is used as audio features. Then the hierarchical Dirichlet process is used to mine their potential emotional events.

### 2.2. Video Emotion Recognition Based on Attention Mechanism

Due to the sparsity of emotional expression in the video, people will focus on some key frames in the perception process of a specific video. These key frames can provide more emotional clues and obtain better emotion recognition performance. Kayaoglu and Eroglu Erdem [21] select key frames for video emotion recognition and achieve good performance. Deng et al. [22] propose an attention-based bidirectional LSTM to focus on the most significant human action to recognize emotion. These methods improve the performance of video emotion recognition by focusing on emotion sensitive regions, but they do not consider the dependence between modes. To solve this problem, Gu et al. [23] introduce a hierarchical multimodal structure, which uses attention mechanism and word-level fusion to recognize emotion from text and audio. Xie et al. [24] associate each convolution window with attention-based weights. Wang et al. [25] propose a two-stage attention and two-stage multitask learning framework. In the first stage, the attention mechanism is used to automatically extract and enhance the features of the corresponding region. Next, the bidirectional recurrent neural network and self-attention network are used to adaptively make full use of the relationship of different levels. CACA-RNN cascade architecture [26] processes face and context information by two RNNs. Both RNNs adopt an attention mechanism; context RNN is used to learn context time information; and face RNN is used to learn face information. Context RNN stores context cues in LSTM neurons to initialize the first time step state of facial RNN. Facial RNN learns facial features and processes context information through an attention mechanism. The output of the last frame of facial RNN is used to recognize video emotion.

The article "Region Dual Attention-Based Video Emotion Recognition" was published in 2022. Journal: Comput Intell Neurosci.

The attention mechanism in this paper not only focuses on key frames in the video but also focuses on the emotion-significant regions in the video frame. The methods [21, 22] mainly focus on key frames, and the significant regions in the video frame have not been considered. In terms of emotional relationship modeling, the existing methods [19, 20, 25, 26] mainly consider the emotional relationship between different modes. This paper mainly focuses on the relationship between different regions of the video frames.

## 3. The Region Dual Attention Based Video Emotion Recognition Method

In this section, the region dual attention-based video emotion recognition method (RDAM) will be introduced in detail. Firstly, the system architecture of the RDAM will be introduced, and then each module of the RDAM will be introduced in detail.

### 3.1. RDAM Architecture

Different regions of video frames contain different emotional cues and play different roles in judging video emotion. In addition, the emotional cues between different regions are often related to each other. Modeling the relationship between different regions will help human emotion recognition. These two aspects are often ignored by the existing video emotion recognition methods. To solve these two problems, a video emotion recognition method based on region dual attention is proposed. It can effectively aggregate the emotional features of different regions and establish the emotional relationship between different regions, so as to improve the accuracy of video emotion recognition.

The article "Region Dual Attention-Based Video Emotion Recognition" was published in 2022. Journal: Comput Intell Neurosci.

Given a video *V*={*I*_1_, *I*_2_,…, *I*_*K*_}, where *K* is the number of video frames of the *V* and *I*_*n*_ is the *n*th video frame. RDAM takes as input the video frame sequence {*I*_1_, *I*_2_,…, *I*_*K*_} and generates a distinguishing video emotion representation that can solve the emotional differences of different regions and make full use of the relationship between different regions.

As shown in Figure 2, RDAM is mainly composed of the regional double attention-based video frames feature extraction network and video frame sequences feature fusion network. The region dual attention-based video frame feature extraction network uses two parallel attention networks to model the emotional differences and relationships between different regions.

ResNet-50 CNN structure [27] is used as the basic model of feature extraction. The downsampling operation is removed in the last two residual network modules so that the final feature mapping size is 1/8 of the input video frame. The emotional features extracted by the residual network are input into two parallel attention modules. The emotional features extracted by ResNet-50 CNN first pass through the regional location attention network to generate a score matrix representing the weights of different regions and then recalculate the emotional features according to the score matrix to obtain the emotional features of perceptible emotion sensitive regions. The emotional features extracted by ResNet-50 CNN pass through the regional relational attention network to generate a regional relationship matrix representing the relationship between any two regions and then recalculate the emotional features according to the regional relationship matrix to obtain the emotional features of perceptible regional relationship.

The emotional features of perceptible emotion sensitive regions and perceptible regional relationships are fused and then pass through a small fully connected network to obtain the emotional features of the video frames. The video frames sequence feature fusion network also adopts an attention module to obtain the emotional weight of the video frame sequences, and video frame sequences are fused according to the emotional weight to generate the final emotional feature of the video. Next, we will introduce the regional location attention module, regional relationship attention module, two attention modules fusion network, and video frames sequence feature fusion in detail.

The article "Region Dual Attention-Based Video Emotion Recognition" was published in 2022. Journal: Comput Intell Neurosci.

### 3.2. Regional Location Attention Module

Each region of high-level features can be regarded as the response of a specific region of the video frame. The responses of all regions of the video frame together constitute the feature of the video frame. However, due to the different emotional sensitivity in different regions, humans often focus on the sensitive regions when judging the emotion of a video frame. For example, given a video frame containing humans, we often recognize human emotion by focusing on the emotional sensitive regions (such as faces) of the human. The emotion recognition method of focusing on local regions is often ignored by deep-learning-based emotion recognition. The emotional sensitivity of different regions is different. To make full use of the emotional sensitive region, meanwhile, the robustness of other regions of the video frame can also be used. This paper proposes a regional location attention module to model the emotional differences of different regions to further improve the ability of emotional feature representation.

After the feature extraction module extracts the features using conv1 to res5c of ResNet-50 CNN, the emotional features of the video frame *M* ∈ *ℜ*^*C*×*H*×*W*^ are obtained. *M* is divided into *H* ∗ *W* regions. Thus, each video frame *I*_*n*_ can be expressed as {*f*_*nl*_}_*l*=1,2,…,*L*_, where *L* = *H* ∗ *W* represents the number of regional features, and each regional feature can be expressed as a *C*-dimensional feature vector, and *l* represents the region number, and it can be expressed as follows:

(1) $$\begin{array}{c} l=\left(i-1\right)\times M+j, \end{array}$$

where *i*=1,2,…, *H*, *j*=1,2,…, *W*.

The regional location attention module generates a regional emotion score for each region. Given an intermediate layer representation *M*, it is first input into a convolution layer to generate a feature map *X*, where *X* is a *H* × *W* matrix. The regional location attention matrix is calculated with the softmax layer, and it can be expressed as follows:

(2) $$\begin{array}{c} x_{ij}=\frac{\exp\left(x_{ij}\right)}{\sum_{i=1}^{H}\sum_{j=1}^{W}\exp\left(x_{ij}\right)}, \end{array}$$

where *x*_*ij*_ indicates the relative importance of the region 〈*i*, *j*〉. The greater the value *x*_*ij*_, the more important the region is.

After obtaining the regional location attention score matrix, the emotional feature *M* is recalculated according to the matrix, and the formula can be expressed as follows:

(3) $$\begin{array}{c} M\left[:,i,j\right]=\frac{M\left[:,i,j\right]\times x_{ij}}{\sum_{i=1}^{H}\sum_{j=1}^{W}x_{ij}}. \end{array}$$

When the emotion features are recalculated according to the regional location attention score matrix, the emotion features that can perceptible emotion sensitive regions are obtained.

The article "Region Dual Attention-Based Video Emotion Recognition" was published in 2022. Journal: Comput Intell Neurosci.

### 3.3. Regional Relationship Attention Module

Distinctive feature representation is very necessary for video emotion recognition. Building the regional relationship attention module to model the relationship between different regions can further improve the ability of regional feature fusion. Thus, the ability of video emotion expression can be enhanced. Next, we will introduce the regional relationship attention network in detail.

As shown in Figure 3, the emotional feature *M* extracted by ResNet-50 CNN is input into two convolution layers, and two mappings B and C are obtained, where B and C are both *H* × *W* matrices. Their dimensions are readjusted to *N* × 1 and 1 × *N*, respectively, where the value of *N* is *H* × *W*. B multiplied by *C* is *S*; then the regional relationship attention matrix is calculated by a softmax layer. The formula can be expressed as follows:

(4) $$\begin{array}{c} s_{ij}=\frac{\exp\left(s_{ij}\right)}{\sum_{i=1}^{N}\sum_{j=1}^{N}\exp\left(s_{ij}\right)}, \end{array}$$

where *s*_*ij*_ indicates the influence of the area *j* on the area *i*. It reflects the importance of emotion recognition when the two regions are fused. The higher the value *s*_*ij*_, the higher the performance improvement when two regions are fused.

After obtaining the regional relationship attention matrix, the emotion features can be recalculated according to the matrix. For each regional feature, it is fused with other regions according to the relationship between the region and other regions. The fused features fully reflect the relationship between different regions. For regional feature 〈*i*, *j*〉, its feature recalculated according to the regional relationship attention matrix can be expressed as follows:

(5) $$\begin{array}{c} M_{ij}^{r}=M_{ij}+\frac{\sum_{h=1}^{H}\sum_{w=1}^{W}M_{hw}\times s_{l\left(i,j\right)l\left(h,w\right)}}{\sum_{h=1}^{H}\sum_{w=1}^{W}s_{l\left(i,j\right)l\left(h,w\right)}}, \end{array}$$

where *l*(*i*, *j*) represents the *l* − th region determined by the value of *i* and *j*. *M*_*ij*_^*r*^ is the recalculated feature of region 〈*i*, *j*〉, which can perceptible regions correlation, according to the region relationship matrix. It reflects the relationship between different regions, and the complementarity between different regions can be guaranteed. The coordination and consistency between different regions are ensured and make the expression of emotional features more effective.

### 3.4. Attention Module Fusion

To make full use of the emotional features of different regions, the features obtained by two parallel attention modules are fused. Specifically, first, the outputs of the two attention modules are transformed by a convolution layer. Let *M*_*n*_^*p*^ be the emotion feature of the video frame *I*_*n*_ output by the regional location attention network, and *f*_*n*_^*p*^ represents the transformed feature of *M*_*n*_^*p*^; *f*_*n*_^*p*^ can be expressed by

(6) $$\begin{array}{c} f_{n}^{p}=\tanh\left(W_{n}^{p}\times M_{n}^{p}+b_{n}^{p}\right), \end{array}$$

where *W*_*n*_^*p*^ and *b*_*n*_^*p*^ are weight parameters. Similarly, let *M*_*n*_^*r*^ be the emotion feature of the video frame *I*_*n*_ output by the regional relationship attention network, and *f*_*n*_^*r*^ represents the transformed feature of *M*_*n*_^*r*^, *f*_*n*_^*r*^ can be expressed by

(7) $$\begin{array}{c} f_{n}^{r}=\tanh\left(W_{n}^{r}\times M_{n}^{r}+b_{n}^{r}\right), \end{array}$$

where *W*_*n*_^*r*^ and *b*_*n*_^*r*^ are weight parameters.

The article "Region Dual Attention-Based Video Emotion Recognition" was published in 2022. Journal: Comput Intell Neurosci.

Then, the corresponding elements of the two features are summed, and the fusion features *f*_*n*_ are obtained through a full connection layer. It should be pointed out that the regional dual attention module is very simple. It can be directly inserted into the existing full convolution network pipeline without adding too many parameters and can effectively enhance the feature representation.

### 3.5. Video Frame Sequences Feature Fusion Network

After obtaining the emotional features *f*_*n*_ of the video frame *I*_*n*_, the video frame sequence feature fusion network fuses features of the video frame sequence {*I*_1_, *I*_2_,…, *I*_*K*_} to generate the emotional features of the video Vmmc5. The network also uses an attention module to obtain the emotional sensitive region of the video frame sequence. Let matrix *F* be the feature set of *K* video frame sequences.

(8) $$\begin{array}{c} F=\left(f_{1},f_{2},\ldots ,f_{K}\right). \end{array}$$

After *F* passes through the attention network of the video frame sequences, the emotional feature representation of video *V* can be obtained:

(9) $$\begin{array}{c} G\left(F\right)=\left(\alpha_{1}f_{1},\alpha_{2}f_{2},\ldots ,\alpha_{K}f_{K}\right), \end{array}$$

where *α*_*i*_ is the weight value of the *i* − th video frame, which represents the emotional weight of the video frame. It can be obtained by learning a linear mapping *W*_*i*_^*g*^ and can be calculated by the following formula:

(10) $$\begin{array}{c} \alpha_{i}=W_{i}^{g}X_{i}, \end{array}$$

where *W*_*i*_^*g*^ is a small fully connected network. In our experiments, two continuous full connection layers are used, and the last full connection layer contains only one neuron.

The article "Region Dual Attention-Based Video Emotion Recognition" was published in 2022. Journal: Comput Intell Neurosci.

The features of different video frames are aggregated according to the emotion weight to obtain the final emotion representation of the video. The aggregation method is as follows:

(11) $$\begin{array}{c} F_{V}=\frac{\sum_{i=1}^{K}\alpha_{i}f_{i}}{\sum_{i=1}^{K}\alpha_{i}}, \end{array}$$

where *F*_*V*_ is the emotional feature of video *V*, and then the emotional feature is passed through a full connection layer and supervised by a softmax loss function.

## 4. Experiments

### 4.1. Video Emotion Recognition Data Set

We conduct experiments on five publicly available video emotion recognition data sets, namely the MHED data set [28], the HEIV data set [29], the ekman-6 data set [30], the videoemotion-8 data set [31], and the SFEW data set [32]. The MHED data set is composed of 1,066 videos that are manually downloaded from the network, and it uses a training set of 638 videos and a testing set of 428 videos. It uses 6 emotion categories “anger,” “disgust,” “fear,” “joy,” “sadness,” and “surprise,” defined by the psychologists Ekman and Friesen [33] to label human emotions in the video. The HEIV data set is composed of 1,012 videos with 607 training videos and 405 for testing. Of the 1,012 annotated videos, 64% are males, and 36% are females. Their ages are distributed as follows: 10% children, 11% teenagers, and 79% adults. Six emotion categories “anger,” “disgust,” “fear,” “joy,” “sadness,” and “surprise,” defined by the psychologists Ekman and Friesen [33], as well as neutral emotion, are used to label human emotions in the video.

The Ekman-6 data set contains 1,637 videos that are manually annotated by 10 annotators according to Ekman's theory [33] on 6 basic human emotion categories. It uses a training set of 819 videos and a testing set of 818 videos with a minimum of 221 videos per category. The VideoEmotion-8 data set contains 1,101 videos collected from YouTube and Flickr with 734 training videos and 367 for testing. The average duration of videos is 107 seconds.

SFEW data set contains over 2,000 minutes of video data that are annotated with valence and arousal values. Similar to [32], we apply an 8:1:1 data set partition.

### 4.2. Ablation Studies

In this subsection, we perform detailed ablation studies on the MHED data set and the HEIV data set to understand the contributions of the proposed model components.

#### 4.2.1. Experimental Results on the MEHD Data Set

To evaluate the regional dual attention module, video frames of the MEHD data set are first extracted, and then the faces of video frames are extracted. Video frames sequence and faces sequence are constructed and are called MEHD-I and MEHD-F, respectively. This subsection will evaluate the regional dual attention network on the video frame sequence MEHD-I and face sequence MEHD-F.

The article "Region Dual Attention-Based Video Emotion Recognition" was published in 2022. Journal: Comput Intell Neurosci.

The regional dual attention network is implemented based on ResNet-50 network to solve the emotional differences of different regions and make full use of the relationship between different regions, to further improve the performance of video emotion recognition. To verify the performance of the regional dual attention module, experiments with different settings were carried out (as shown in Table 1).

As shown in Table 1, the regional dual attention module improves the performance of video emotion recognition. The emotion recognition accuracy using the regional location attention module is 46.73%, and the accuracy is improved by 2.57% compared with the benchmark model ResNet-50. Meanwhile, the accuracy of using the regional relationship attention mechanism is improved by 2.1% compared with the benchmark model ResNet-50. When the two attention modules are combined, the performance is improved by 3.27%. The experimental results show that the regional dual attention module is very helpful to the performance of video emotion recognition.

Next, experiments are carried out on the face sequence MEHD-F to further verify the effectiveness of our method (as shown in Table 2). The recognition accuracy of the benchmark model ResNet-50 is 52.34%. The emotion recognition accuracy is 58.88% using the regional location attention module alone, and the accuracy is improved by 6.54%. Meanwhile, the accuracy of using the regional relationship attention mechanism alone is 6.07% higher than ResNet-50. When the two attention modules are combined, the performance is improved by 7.47%. The existing attention mechanism mainly models the emotional differences between different video frames and improves the performance by effectively fusing the emotional features of different video frames. Different from the existing methods, the regional location attention mechanism and regional relationship attention mechanism model the emotional differences between different regions of the same video frame, so as to make full use of the differences in emotion expression between different regions to improve the performance of emotion recognition.

#### 4.2.2. Experimental Results on HEIV Data Set

In this subsection, we conduct experiments on HEIV data sets to further evaluate the effectiveness of the RDAM method. Similar to the MEHD data set, video frames of the HEIV data set are first extracted, and then the faces of the video frames are extracted. Video frames sequence and faces sequence are constructed and are called HEIV-I and HEIV-F, respectively. This subsection will evaluate the regional dual attention network on the video frame sequence HEIV-I and face sequence HEIV-F.

The article "Region Dual Attention-Based Video Emotion Recognition" was published in 2022. Journal: Comput Intell Neurosci.

Table 3 shows the experimental results on the HEIV-I. The recognition accuracy of the benchmark model ResNet-50 is 42.22% on the HEIV-I data set. The accuracy using the regional location attention module alone is 44.69%, and the accuracy is improved by 2.47%. Meanwhile, the accuracy of using the regional relational attention mechanism alone is improved by 1.97%. When the two attention modules are combined, the performance is improved by 3.47%.

Table 4 shows the experimental results on the HEIV-F. The recognition accuracy of the benchmark model ResNet-50 is 44.94% on the HEIV-F data set. The accuracy using the regional location attention module alone is 49.38%, and the accuracy is improved by 4.44%. Meanwhile, the accuracy of using the regional relational attention mechanism alone is improved by 4.2%. When the two attention modules are combined, the performance is improved by 5.18%.

### 4.3. Comparison with State of the Art

In this subsection, we compare the state-of-the-art performance in recent literature. MHED-I and MHED-F are video frames sequence and faces sequence, respectively. The above evaluation is from the perspective of single mode. The experimental results show that both the regional location attention module and the regional relationship attention module can improve the accuracy of emotion recognition. Most of the existing video emotion recognition methods use multimodal feature fusion. To evaluate the performance of the proposed method, the performance is compared with the existing methods on the MHED data set and the HEIV data set. The video frames and facial features of the MHED data set and the HEIV data set are extracted, respectively, and these two features are fused to obtain the final emotional representation of the video.  Table 5 gives top-1 accuracy (%) of different methods on the MHED and HEIV data sets. Quality-aware network (QAN) is mainly used to solve the quality difference between images. The accuracy of QAN that only takes images as input is the lowest. The accuracy of QAN on the MHED and HEIV data sets is 46.03% and 43.95%, respectively. The performance of multimodal features fusion literature [12] and spatial-temporal feature fusion network [13] are all better than QAN. This is because a multimodal features' fusion network, which uses multiple modes can achieve better performance. Attention Clusters [7] are used to extract the fc6 layer features of faces, scenes, and images of videos, and then they are sent to an attention network. Features of each modal are aggregated according to the output of the attention network, and the emotion feature of each modal is produced. Finally, features of the three modes are concatenated and passed a fully connected layer and are supervised by softmax loss, and the final emotion feature of the video is produced. The accuracy of the attention cluster on the MHED and HEIV data sets is 59.81% and 49.63%, respectively. The performance of the attention clusters is better than those feature fusion methods without an attention mechanism. Our RDAM achieves 6.08% and 3.46% top-1 performance gain on the MHED and HEIV data sets. Note that our work attains superior performance for two reasons: firstly, the regional location attention mechanism can make full use of the emotional differences of different regions. Secondly, the regional relationship attention mechanism can make full use of the relationship between different regions.

The article "Region Dual Attention-Based Video Emotion Recognition" was published in 2022. Journal: Comput Intell Neurosci.

To further evaluate the effectiveness of our method, we also conduct experiments on the Ekman-6 and VideoEmotion-8 data sets.  Table 6 gives top-1 accuracy (%) of different methods on the Ekman-6 and VideoEmotion-8 data sets. As shown in Table 6, our RDAM achieves a 3.06% and 2.45% performance gain on the Ekman-6 and VideoEmotion-8 data sets, respectively. The emotion in context [12] only fuses context information, and it has the lowest accuracy. Xu et al. [30] further improve the performance by transferring knowledge from heterogeneous external sources. The frame relationships or regions of interest are studied in the papers [34] (Kernelized feature) and [35] (concept selection), and the accuracy is further improved. The accuracy of graph-based network on the Ekman-6 and VideoEmotion-8 data sets is 55.01% and 51.77%, respectively. It utilizes the semantic relationships of different regions based on the graph convolutional network [36] to improve performance. The results show that our method achieves the state-of-the-art results on both Ekman-6 and VideoEmotion-8 data sets. This is because our method addresses the problem of the emotional differences between different regions and can make full use of the relationship between different regions.

On SFEW, we compare against RAN [37], DDL [38], and FDRL [39].  Table 7 shows the results. Among all the competing methods, RAN and DDL aim to disentangle the disturbing factors. These methods improve the performance by reducing the effect of different disturbing factors, but they ignore large expression similarities among different expressions. FDRL views the expression information as the combination of the shared information across different expressions and the unique information for each expression. In contrast, our method solves the emotional differences of different regions and makes full use of the relationship between different regions.  Table 7 shows the effectiveness of our proposed method.

The article "Region Dual Attention-Based Video Emotion Recognition" was published in 2022. Journal: Comput Intell Neurosci.

## 5. Conclusions and Future Work

In this paper, a region dual attention-based video emotion recognition method (RDAM) is proposed to effectively solve the emotional differences between different regions and make full use of the relationship between different regions. Specifically, RDAM is composed of two parallel attention modules: one is the regional location attention module, which generates a score matrix representing the weights of different regions and then recalculates the emotional features according to the score matrix to obtain the features of perceptible emotional sensitive regions. The other is the regional relationship attention module, which generates a regional relationship matrix representing the relationship between any two regions, and then the emotional features are recalculated according to the regional relationship matrix to obtain the emotional features that can perceptible regions correlation. The two features are fused to obtain the emotional features of video frames. Finally, the attention-based video frame sequence feature fusion network is used to fuse the video frame sequence, and the emotional feature of the video is obtained. A series of experiments are carried out on four public video emotion recognition data sets. The experimental results show that RDAM can effectively solve the emotional differences between different regions and make full use of the relationship between different regions, to improve the performance of emotion recognition. In addition, it is very important to reduce the computational complexity and enhance the robustness of the model. In the next step, we will study how to reduce the computational complexity and improve the robustness while ensuring performance.

## Figures and Tables

**Figure 1:** Motivation of the region dual attention-based video emotion recognition model.

**Figure 2:** Framework of the region dual attention-based video emotion recognition model.

**Figure 3:** Region relationship attention module.

**Table 1:** Evaluation of region dual attention mechanism on MHED-I data set.

Method	Accuracy (%)
ResNet-50 + average aggregation	44.16
ResNet-50 + regional location attention mechanism	46.73
ResNet-50 + regional relationship attention mechanism	46.26
ResNet-50 + regional dual attention mechanism	47.43

**Table 2:** Evaluation of region dual attention mechanism on the MHED-F data set.

Method	Accuracy (%)
ResNet-50 + average aggregation	52.34
ResNet-50 + regional location attention mechanism	58.88
ResNet-50 + regional relationship attention mechanism	58.41
ResNet-50 + regional dual attention mechanism	59.81

The article "Region Dual Attention-Based Video Emotion Recognition" was published in 2022. Journal: Comput Intell Neurosci.

**Table 3:** Evaluation of region dual attention mechanism on the HEIV-I data set.

Method	Accuracy (%)
ResNet-50 + average aggregation	42.22
ResNet-50 + regional location attention mechanism	44.69
ResNet-50 + regional relationship attention mechanism	44.19
ResNet-50 + regional dual attention mechanism	45.68

**Table 4:** Evaluation of region dual attention mechanism on the HEIV-F data set.

Method	Accuracy (%)
ResNet-50 + average aggregation	44.94
ResNet-50 + regional location attention mechanism	49.38
ResNet-50 + regional relationship attention mechanism	49.14
ResNet-50 + regional dual attention mechanism	50.12

**Table 5:** Top-1 accuracy (%) compared with related works on the MHED and HEIV.

Method	Accuracy on MEHD (%)	Accuracy on HEIV (%)
Quality-aware network [6]	46.03	43.95
Vielzeuf et al. [13]	53.73	45.93
Chen et al. [12]	55.60	46.17
Attention clusters [7]	59.81	49.63
Our method	65.89	53.09

**Table 6:** Top-1 accuracy (%) comparing with state-of-the-art methods on Ekman-6 and VideoEmotion-8.

Method	Ekman (%)	VideoEmotion-8 (%)
Emotion in context [12]	51.8	50.6
Xu et al. [30]	50.4	46.7
Kernelized feature [34]	54.4	49.7
Concept selection [35]	54.40	50.82
Graph-based network [36]	55.01	51.77
Ours	58.07	54.22

We also evaluate the performance of our method on the SFEW data set for cross-validation purposes.

**Table 7:** Top-1 accuracy (%) compared with state-of-the-art methods on SEWA.

Method	SFEW (%)
RAN [37]	56.40
DDL [38]	59.86
FDRL [39]	62.16
Ours	63.41

## Data Availability

Ekman-6 and VideoEmotion-8 are two public data sets. MHED and HEIV data sets can be obtained from the corresponding author upon request.
